The article "Study of the Relationship between Microbiome and Colorectal Cancer Susceptibility Using 16SrRNA Sequencing" was published in 2020. Journal: Biomed Res Int.

# Study of the Relationship between Microbiome and Colorectal Cancer Susceptibility Using 16SrRNA Sequencing

**DOI:** 10.1155/2020/7828392

**Published:** 2020-01-30

**Authors:** Wanxin Liu, Ren Zhang, Rong Shu, Jinjing Yu, Huan Li, Hui Long, Shu Jin, Shengbao Li, Qiuyu Hu, Fei Yao, Chuanren Zhou, Qiyou Huang, Xiafen Hu, Meng Chen, Weiguo Hu, Qiang Wang, Shenying Fang, Qingming Wu

**Affiliations:** ^1^Institute of Infection, Immunology and Tumor Microenvironment, Hubei Province Key Laboratory of Occupational Hazard Identification and Control, Medical College, Wuhan University of Science and Technology, Wuhan 430065, China; ^2^Department of Anesthesiology, The Third People's Hospital of Hubei Province, Wuhan 430030, China; ^3^Department of Gastroenterology, Tianyou Hospital, Wuhan University of Science and Technology, Wuhan, Hubei, China; ^4^Department of Gastroenterology, Taihe Hospital, Hubei University of Medicine, Shiyan, Hubei, China; ^5^Department of Oncology, Renmin Hospital of Wuhan University, Wuhan 430060, China

## Abstract

A lot of previous studies have recently reported that the gut microbiota influences the development of colorectal cancer (CRC) in Western countries, but the role of the gut microbiota in Chinese population must be investigated fully. The goal of this study was to determine the role of the gut microbiome in the initiation and development of CRC. We collected fecal samples of 206 Chinese individuals: 59 with **polyp** (group P), 54 with **adenoma** (group A), 51 with **colorectal cancer** (group CC), and 42 **healthy controls** (group HC).16S ribosomal RNA (rRNA) was used to compare the microbiota community structures among healthy controls, patients with polyp, and those with adenoma or colorectal cancer. Our study proved that intestinal flora, as a specific indicator, showed significant differences in its diversity and composition. Sobs, Chao, and Ace indexes of group CC were significantly lower than those of the healthy control group (CC group: Sobs, Chao, and Ace indexes were 217.3 ± 69, 4265.1 ± 80.7, and 268.6 ± 78.1, respectively; HC group: Sobs, Chao, and Ace indexes were 228.8 ± 44.4, 272.9 ± 58.6, and 271.9 ± 57.2, respectively). When compared with the healthy individuals, the species richness and diversity of intestinal flora in patients with colorectal cancer were significantly reduced: PCA and PCoA both revealed that a significant separation in bacterial community composition between the CC group and HC group (with PCA using the first two principal component scores of PC1 14.73% and PC2 10.34% of the explained variance, respectively; PCoA : PC1 = 14%, PC2 = 9%, PC3 = 6%). Wilcox tests was used to analyze differences between the two groups, it reveals that *Firmicutes* (*P*=0.000356), *Fusobacteria* (*P*=0.000001), *Proteobacteria* (*P*=0.000796), *Spirochaetes* (*P*=0.013421), *Synergistetes* (*P*=0.005642) were phyla with significantly different distributions between cases and controls. The proportion of microorganism composition is varying at different stages of colon cancer development: *Bacteroidetes* (52.14%) and *Firmicutes* (35.88%) were enriched in the healthy individuals; on the phylum level, the abundance of *Bacteroidetes* (52.14%-53.92%-52.46%–47.06%) and *Firmicutes* (35.88%-29.73%-24.27%–25.36%) is decreasing with the development of health-polyp-adenomas-CRC, and the abundance of *Proteobacteria* (9.33%-12.31%-16.51%–22.37%) is increasing. PCA and PCOA analysis showed there was no significant (*P* < 0.05) difference in species similarity between precancerous and carcinogenic states. However, the composition of the microflora in patients with precancerous lesions (including patients with adenoma and polyp) was proved to have no significant disparity (*P* < 0.05). Our study provides insights into new angles to dig out potential biomarkers in diagnosis and treatment of colorectal cancer and to provide scientific advice for a healthy lifestyle for the sake of gut microbiota.

## 1. Introduction

Colorectal cancer (CRC) has been a common malignancy all around the world; colorectal cancer (CRC) is the second leading cause of cancer death and is the third most common malignancy in the world [1]. Global epidemiological characteristics show that the global burden of colorectal cancer (CRC) is expected to increase by 60% by 2030, with more than 2.2 million new cases and 1.1 million deaths [2]. In China, the urban cancer screening program included more than 1.38 million people, of whom 182,927 were assessed to be at high risk for colorectal cancer (CRC) [3].

There is increasing evidence that gut microbiota contributes to the carcinogenesis of colorectal cancer (CRC) [4], along with genetic and other factors [5], including age, sex, family history, excessive alcohol consumption, diets [6] with high animal fat, and diets low in fruit and vegetable fiber. The intestinal flora is more like one of our organs, providing a new pathway for therapeutic intervention as well as a part of the immune system, supporting the host to promote health or initiate disease [7]. Microbiota, associated with the human body, also play a role in shaping the inflammatory environment and promoting tumor growth and spread [8].

The role for microorganisms that initiate and facilitate the process of colorectal cancer has become clear [9]. Global data revealed the characteristic flora of colorectal cancer, and 29 species were found to have increased abundance in the fecal flora of patients with colorectal cancer (CRC) [10]. The microflora is involved in the initiation, development, and spread of tumor. Recently, it has become increasingly clear that microflora, especially intestinal microflora, can regulate the response to tumor treatment and the sensitivity to toxic and side effects [11].

Along with the evolution of gut microbiota, some researchers have hypothesized that modulating the microbiota could be a lead for new targeted therapy [12]. As a very prevailing therapy, microbiome-targeted therapy or cancer bacteriotherapy were designed based on how to modulate gut microbiota with a change of diet, probiotics, and fecal transplantation. The effectiveness and safety of microflora transplantation for tumor treatment is the core issue in this field of translational research. Colon tumors were the first to benefit from it [13].

Here, we perform 16S ribosomal RNA (rRNA) gene sequencing on fecal microbiome of normal colorectal individual, polyp, adenoma and adenocarcinomas. The gut microbiota, either as individual microbes or as a microbial community exerting a collective effect, may promote or mitigate the stages of colorectal carcinogenesis [14], and we have confirmed it in animal studies as well.

What we are trying to achieve is that the characteristics and functions of CRC-related microflora are expected to be used in the diagnosis and treatment of CRC worldwide, and certain valuable “gut advices” can be put forward to human health.

## 2. Materials and Methods

### 2.1. Sampling

A case-control study was conducted in Tianyou hospital affiliated to Wuhan University of Science and Technology between January 2017 and December 2017. We surveyed individuals who had undergone standardized colonoscopic examinations and physical examinations at the hospital and enrolled 206 individuals as our research objects.

#### 2.1.1. CRC Patients (*n* = 51)/Polyps (*n* = 59)/Adenomas (*n* = 54)/Healthy Control (*n* = 42)

Individuals who visited the department of gastroenterology of Tianyou hospital of Wuhan from January 2017 to December 2017 and received colonoscopy and histopathological examination were recruited to the study. At the same time, healthy volunteers were recruited as the health control group in Wuhan University of science and technology. The subjects were divided into four groups, and among them, patients with colorectal adenocarcinoma were recorded as the colorectal cancer (CC) group, patients with colorectal adenoma were recorded as the adenoma (A) group, and patients with colorectal polyps were recorded as the polyp (P) group. The recruited healthy control population was recorded as the healthy control (HC) group. Exclusion criteria were a personal history of CRC, IBD, or IBS (see Table 1).

#### 2.1.2. Ethics Statement

The study was approved by the hospital ethics committee, and all subjects signed informed consent.

### 2.2. Methods

#### 2.2.1. Sample Collection and Preservation

Objects were collected in the clean environment of fresh feces (not less than 6 g), put in an aseptic sampling tube and sent to the laboratory, and kept at −80°C for inspection. Stool samples were collected before surgery and electronic colonoscopy in patients with rectal cancer, adenoma, and polyp, and during the collection process, the samples should not be contaminated by urine or sewage.

#### 2.2.2. DNA Extraction and Amplification of 16S rRNA Gene Fragment

DNA from the stool sample is extracted by referring to the instructions given by the QIAamp DNA Stool Mini Kit, DNA concentration is determined, and stored at −20°C for further analysis.

The variable region of 16S rDNA gene V4 was amplified by PCR and primers 515F5′-GTGCCAGCMGCCGCG GTAA-3′ and 806R 5′-GGACTACHVGGGTWTCTAAT-3′ (Table 2).

Amplification conditions were as follows: 95°C solution chain for 2 min, 95°C, 30 s, 30 s, 55°C 72°C 45 s, 25 cycles, and 72°C extending for 5 min.

Illumina MiSeq sequencing: PCR products were recovered after 2% agarose gel electrophoresis, purified using AxyPrep DNA gel recovery kit instructions, and quantified using the quantitatively fluorescent-st blue fluorescence quantitative system. The purified amplicon was mixed proportionally according to the required sequencing quantity and sent to the BGI company (Wuhan of Hubei, China) for high-throughput sequencing on the Illumina MiSeq platform.

#### 2.2.3. Analysis of Community Patterns

The tags were clustered to OTU (Operational Taxonomic Unit) by scripts of software USEARCH (v7.0.1090) [15]. Databases used for species annotation: 16S rDNA is used for bacterial and archaea community: Greengene (default): V201305 [16]; RDP: Release9 201203 [17].

OTUs were filtered as follows:

1. Unassigned OTUs were removed.
2. OTUs not assigned to the target species were removed. For example, the OTUs assigned to archeae would be removed if the project is about 16S rDNA for bacterial community study.

#### 2.2.4. Cluster Analysis of OTU

Operational Taxonomic Units (OTUs) are markers of a group derived from a Taxonomic unit (strain, genus, species, grouping, etc.) in the study of phylogeny or population genetics, with the purpose of simplifying analysis. In this study, OTU represents the sequence from the same source. Uparse software was used to perform OTU clustering on the above-processed Clean Tags with 97% similarity, and Uchime 4.2 was used. The software was compared with the existing 16S chimera database gold database, and the chimera generated by PCR amplification in the OTU sequence was removed.

#### 2.2.5. OTU Venn Chart

Venn diagram could visually display the number of common/unique OTUs in multisamples/-groups. The core microbiomes of different environments could be obtained if combined with the OTU representing species. Based on the OTU abundance, OTU of each group was listed and Venn diagram was drawn by Venn Diagram of software R (v3.1.1).

#### 2.2.6. OTU PCA Analysis

In order to display the differences of OTU composition in different samples, principal component analysis (PCA) was used to construct a 2D graph to summarize factors mainly responsible for this difference, and similarity is high if two samples are closely located. Based on the OTU abundance information, the relative abundance of each OTU in each sample will be calculated, and the PCA of OTU was done with the relative abundance value. The software used in this step was package “ade4” of software R (v3.1.1).

#### 2.2.7. OTU Rank Curve

The OTU rank abundance curve provides a means for visually representing species richness and species evenness. Species richness can be viewed as the number of different species on the chart (*x*-axis), i.e., how many species were ranked. Species evenness is derived from the slope of the line that fits the graph. A steep gradient indicates low evenness as the high ranking species have much higher abundances than the low ranking species. A shallow gradient indicates high evenness as the abundances of different species are similar. OTU were ranked by the relative abundance value as *x*-axis and the OTU relative abundance as *y*-axis; then, the rank curve was drawn by software R (v3.1.1).

#### 2.2.8. Species Annotation

The tag number of each taxonomic rank (Phylum, Class, Order, Family, Genus, and Species) or OTU in different samples were summarized in a profiling table or histogram, and the histogram was drawn with the software R (v3.1.1).

Based on Greengene database (V201305), RDP classifer 2.2 software Bayesian algorithm is used to compare the representative sequences of each OTU obtained with the database for similarity and species annotation and to calculate the community composition of each sample at various classification levels of phylum, class, order, family, genus, and species and visualized with a histogram.

#### 2.2.9. Diversity Analysis with Single Sample

Alpha diversity is applied for analyzing complexity of species [18] diversity for a sample through several indices, including observed species, Chao1, Ace, Shannon, and Simpson. The complexity of the sample is proportional to the first four values, with a negative correlation with the Simpson value. Observed species value, Chao1 value, and Ace value can reflect the species richness of the community.

The Shannon value and Simpson value can reflect the species diversity of the community, affected by both species richness and species evenness, that is, the two values also consider the abundance of each species. With the same species richness, the greater the species evenness, the greater the community diversity.

#### 2.2.10. Rarefaction Curve

The indices are calculated by Mothur (v1.31.2), and the corresponding rarefaction curve is drawn by software R (v3.1.1).

The rarefaction curve based on the three values could also be used to evaluate if produced data is enough to cover all species in the community. When the curve tends to be smooth, it suggests the produced data are enough. Otherwise, when the curve continues to climb with increasing sequencing effort, it shows a high complexity in samples, and there still will be species uncovered by the sequencing data.

#### 2.2.11. Diversity Analysis among Samples (*n* ≥ 4)

Beta diversity analysis was used to evaluate differences of samples in species complexity. Beta diversity analysis was performed by software QIIME (v1.80).

Various values, such as Bray–Curtis, weighted UniFrac, unweighted UniFrac, and Pearson, could be used to measure beta diversity, especially the first three values. Bray–Curtis distance is a commonly used index to reflect the differences between two communities, and UniFrac uses the system evolution information to compare the composition of community species between samples.

The results can be used as a measure of beta diversity. It takes into account the distance of evolution between the species, and the bigger the index is, the greater are the differences between samples.

#### 2.2.12. Principal Coordinates Analysis

Principal coordinates analysis (PCoA) is a multivariate statistical analysis method that selects a few important elements from several influencing factors through linear transformation, reduces dimensionality of multidimensional data to extract the most important elements, and visually presents the results in a two-dimensional coordinate graph to reflect differences between groups.

By using iterative algorithm in QIIME1.8 software, PCoA analysis was carried out based on the beta-diversity index matrix obtained by the abovementioned calculation, and the main coordinate with the largest contribution rate was selected to draw the coordinate diagram.

In the coordinate graph, the closer the distance between the two samples is, the more similar is the species composition of the two samples, so that the differences in species composition and structure of the samples can be observed.

#### 2.2.13. Significant Differences Analysis between Groups of Samples (Groups ≥ 2, Samples per Group ≥ 3)

We use the method of statistical analysis to get the abundance differences of microbial communities between samples, and FDR (false discovery rate) is adopted to assess the significance of differences.

Metastats and R (v3.1.1) are used to determine which taxonomic groups were significantly different between groups of samples. We adjusted the obtained *P* value by a Benjamini–Hochberg false discovery rate correction (function “p.adjust” in the stats package of R (v3.1.1)) [19].

## 3. Result

### 3.1. Dysbiosis in Gut Microbiome Is Closely Related to Colorectal Cancer Susceptibility

#### 3.1.1. OUT Analysis

OTU clustering was carried out for the sequence at 97% similarity, and a total of 2170 OTUs were obtained, with an average of 23 OTUs of each sample. Venn diagram of OUT showed that the healthy control group (HC) obtained a total of 959 OTUs, the CC group owned 1211 OTUs, and two groups share 837 OTUs. The unoverlapped portion represents the number of OTUs is unique to the group. Compared with the HC group, CC group had more unique OTU numbers (see Figure 1(a)).

In addition, the dilution curve of the alpha diversity index (Sobs index) shows the curve flattens out, which indicates the sample sequencing is sufficient, and the sequencing depth is basically covered (see Figure 1(b)). In other words, there are fewer undetected species among the ones we detect, and it guarantees the reliability of our research.

Principal component analysis (PCA) based on the relative abundance of genera revealed a significant separation in bacterial community composition between the CC group and HC group using the first two principal component scores of PC1 and PC2 (14.73% and 10.34% of explained variance, respectively; Figure 1(c)). We also found a certain degree of clustering among some samples, which revealed that the intestinal flora changed to some extent.

Rank charts show two aspects of species diversity: species abundance and species evenness. In the horizontal direction, the width of the curve reflects the abundance of species. The more the curve crosses the horizontal axis, the higher the abundance of species will be. The gentleness of the curve reflects the species uniformity in the sample. The gentler the curve is, the more homogeneous the species distribution is; the steeper the curve is, the more heterogeneous the species distribution is. Compared with the HC group, the transversal range of the CC group was larger, indicating that the species richness was increased. The curve is steep, indicating a decrease in species evenness (see Figure 1(d)).

#### 3.1.2. Alpha Diversity Analysis

Alpha diversity is the analysis of species diversity in samples, and Ace, Chao, Shannon, and Simpson indexes are calculated based on OTU species and abundance. The Sobs, Chao, Ace richness index, Shannon, and Simpson diversity index were used to describe the diversity features of our colorectal community results. Sobs, Ace, and Chao indexes reflect the species richness in the sample, that is, the number of OTU. The Shannon index and Simpson index were used to reflect community diversity, including species richness and species evenness. Therefore, the larger the Shannon index and the smaller the Simpson index, the higher the species diversity in the sample.

As shown in Figure 2, Sobs, Chao, and Ace indexes of group CC were significantly lower than those of the healthy control group. The results showed that species richness of group CC was significantly lower than that of the healthy control group. In addition, the Shannon index of group CC was lower than that of the HC group, and the Simpson index was higher than that of the HC group, but the difference was not statistically significant (Figure 2, Table 3).

#### 3.1.3. Beta Diversity Analysis

In order to further display differences in species diversity among samples, principal coordinates analysis (PCOA) is used to display differences among samples. If the two samples are close together, the species composition of the two samples is similar. A significant separation in bacterial community composition between group HC and group CC is revealed according to the 3d image (Figure 3).

### 3.2. Structure Analysis of the Microbiota Associated with Colorectal Cancer

#### 3.2.1. The Microbial Composition of Groups HC and CC at the Phylum Level

The group HC and group CC contain 11 kinds of bacteria at the level of phylum: *Bacteroidetes*, *Firmicutes*, *Proteobacteria*, *Actinobacteria*, *Fusobacteria*, *Verrucomicrobia*, *Synergistetes*, *Tenericutes*, *Cyanobacteria*, *TM7*, and *Lentisphaerae* (Figure 4).

At the phylum level, each group of samples showed significant individual differences: *Proteobacteria* accounted for 9.3% to 22.4% of the two groups; the proportion of *Fusobacteria* in two groups ranged from 0.6% to 3.4% (Figure 5).

#### 3.2.2. The Microbial Composition of Groups HC and CC at the Genus Level

The two groups contain 13 bacteria at the level of genus: *Bacteroides*, unclassified, *Escherichia*, *Prevotella*, *Sutterella*, *Faecalibacterium*, *Clostridium*, *Streptococcus*, *Parabacteroides*, *Ruminococcus*, *Haemophilus*, *Roseburia*, and *Megamonas* (see Figure 6). The dominant bacteria in the abovementioned samples are listed in Figure 5. In the healthy control group (HC), the dominant bacteria are *Prevotella*, *Bacteroides*, unclassified, *Faecalibacterium*, *Escherichia*, *Roseburia*, and *Megamonas*, and the proportion is 30%, 30%, 13%, 12%, 7%, 4%, and 4%, respectively; in the group CC, the dominant bacteria contain *Bacteroides*, unclassified, *Escherichia*, *Prevotella*, *Sutterella*, and *Faecalibacterium*, and the proportion is 39%, 17%, 15%, 8%, 4%, and 4%, respectively.

#### 3.2.3. Analysis on Composition Difference of Gut Microbiota

Wilcox tests were employed to analyze differences in the abundance between two groups for normally or not normally distributed data, respectively. The differences in microbial community abundance between the two groups were examined by statistical methods, and the significance of the differences was evaluated by FDR (false discovery rate). We screened out the species that caused the difference in the composition of the two groups of samples (see Table 4). *Firmicutes*, *Fusobacteria*, and *Proteobacteria* are the main difference in the phyla.

### 3.3. Internal Causal Relationship between Gut Microbiota and Different Stages of Colorectal Carcinogenesis

According to our existing research findings and combined with accumulated research, there is unequivocal evidence linking gut dysbiosis to CRC development. We identified that the microbial structures of the CRC patients and healthy individuals differed significantly. However, gut dysbiosis and the occurrence of CRC, which occur first, is not yet very clear.

With reference to the clinicopathological staging criteria of colon cancer, we selected all pathological diseases during the development of colon cancer, including health status, polyp, adenoma, and cancer stage, and detailed group information has been mentioned above.

Through 16S ribosomal RNA (rRNA) gene sequence, the unique role of intestinal flora across the whole course of CRC disease was comprehensively analyzed.

#### 3.3.1. Richness and Diversity Analysis

The Chao richness index, Shannon index, and Simpson diversity index were used to describe the alpha diversity features of our bacterial community results. We found that the Chao richness index of the microbiota was significantly different in the 4 groups (Chao richness index for the normal, polyp, adenoma, and cancer group were 271.9 ± 58.6, 238.4 ± 70.1, 240.0 ± 63.2, and 265 ± 80.7, respectively, *P*=0.01818, Figure 7(b)), while the Shannon index and Simpson index in the 4 groups were not significantly different: the Shannon index for the normal, polyp, adenoma, and cancer group was 3.01 ± 0.56, 2.72 ± 0.72, 2.77 ± 0.59, and 2.79 ± 0.77, respectively, *P*=0.1396 (Figure 7(d)), and the Simpson index for normal, adenoma, and cancer groups was 0.14 ± 0.10, 0.18 ± 0.13, 0.15 ± 0.10, and 0.17 ± 0.15, respectively, *P*=0.23747 (Figure 7(e), Table 5).

Principal component analysis (PCA) based on the relative abundance of genera revealed a significant separation in bacterial community composition between group HC and group P using the first two principal component scores of PC1 and PC2 (16.63% and 8.65% of explained variance, respectively, Figure 8(a)). Similarly, a separation sign can be found between group A and group HC using the first two principal component scores of PC1 and PC2 (16.69% and 8.41% of explained variance, respectively, Figure 8(b)), indicating that compared with healthy control, gut microbiota differs between patients with polyp, adenoma, and CRC.

In order to further illustrate the difference between precancerous lesions, including polyp and adenoma, and oncogenous state, principal coordinates analysis (PCoA) is used to display differences among samples. If the two samples are close together, the species composition of the two samples is similar (Figure 9).

When the species similarity was analyzed in combination with the overall development stage of colorectal cancer, there is a new discovery: there was no significant difference in species similarity between precancerous and carcinogenic states (Figure 10).

*Bacteroidetes* and *Firmicutes* were enriched in the healthy control group compared with the polyp, adenoma, and CRC groups (*Bacteroidetes*: 52.14% vs. 53.92% in HC and polyp groups, respectively; 53.92% vs. 52.46% in polyp and adenoma groups, respectively; and 52.46% vs. 47.06% in adenoma and CRC group, respectively; *Firmicutes*: 35.88% vs. 29.73% in HC and polyp groups, respectively; 29.73% vs. 24.27% in polyp and adenoma groups, respectively; and 24.27% vs. 25.36% in adenoma and CRC group, respectively). *Proteobacteria* was relatively scarce in the HC group compared with the other 3 groups (9.33% vs. 12.31% in HC and polyp groups, respectively; 12.31% vs.16.51% in polyp and adenoma groups, respectively; and 16.51% vs. 22.37% in adenoma and CRC group, respectively) (Figures 5, 11, and Table 5).

#### 3.3.2. Taxa Analysis at the Phylum Levels

Based on the analysis of the composition of every group, among all bacteria at the phylum level, the predominant phyla were *Bacteroidetes*, *Firmicutes*, *Proteobacteria*, *Fusobacteria*, and *Actinobacteria*.

There is the trend chart based on the overall microbial composition for each group at the phylum level (Figure 12), and we found that the proportion of microorganism composition is different at different stages of colon cancer development, that is to say, abundance of gut microbial also varies.

### 3.4. Digging for a Distinct Biomarker

The Wilcoxon and Kruskal–Wallis test were conducted in R, and the *P* values were adjusted using the Benjamin–Hochberg method. A Benjamin–Hochberg *P* value <0.05 was considered to be significant.

We screened all groups of statistically significant species, listed in Table 6. When comparing the healthy group and the disease groups, as the specific bacteria, *Fusobacteria* and *Firmicutes* can clearly distinguish the disease group from the healthy group, whether the disease is at the period of polyp, adenoma, or cancer, not only that, with the development of health-adenomas-CRC, health-polyp-adenomas, or health-adenomas-CRC, regardless of the disease progression sequence mentioned above, *Fusobacteria* always exhibits the characteristics of a marker species (Table 7).

## 4. Discussion

This study provides evidence that gut microbiota is closely linked to CRC development. We confirm that the microbiota of patients with CRC differs from that of healthy controls. In our study, we demonstrate that as colorectal neoplasm progresses along the polyp-adenoma-carcinoma sequence, gut microbiota formed a specific structure network with some functional features. The gut microbiota has formed a symbiotic connection with humans that is imperative for life. Wang et al. [20], along with his team, analyzed the stool samples of CRC Chinese patients, and found that *Bacteroides fragilis*, *Enterococcus*, *Escherichia/Shigella*, *Klebsiella*, and *Streptococcus*, and *Peptostreptococcus* displayed a higher relative abundance in CRC patients, while *Roseburia*- and *Lachnospiraceae*-related OTUs dominated high load in the healthy controls. Researchers also concluded that the CRC patients had a lower microbiota diversity and Clostridia abundance, but a high abundance of *Fusobacterium* and *Porphyromonas* at the genus level in another study [21]. *Fusobacterium* was identified to be the most common bacterial species in colorectal cancer tissues and metastases with colorectal cancer cells [22], *Fusobacterium* (an anaerobe in the oral cavity) is associated with colorectal cancer, the abundance of *Fusobacterium* in tumor tissues and feces of patients with colorectal cancer was significantly increased, and the inflammatory response caused by *clostridium nucleate* may also promote the development of colorectal cancer [23]. *Fusobacterium nucleatum* is enriched in colorectal cancer (CRC) tissues and can affect multiple stages of CRC progression: promoting cancer cell proliferation, tumor immune escape, recurrence and chemotherapy resistance, and so on. *Fusobacterium nucleatum* can be used as a potential marker for the diagnosis and prognosis evaluation of CRC and is also a potential target for the treatment of CRC [24–32].

Unlike the other experimental schemes [14, 33], a unique feature of our experimental design is the sampling of individuals at distinct stages of colorectal neoplasia, which covered almost all symbolic precancerous stages. We got the richness and we compared the composition of gut microbiota at each stage, and our systematic analysis draw attention to the importance of microbial consortia as a potential player in colorectal tumor development.

Compared with healthy individuals, *Bacteroidetes*, *Firmicutes*, and *Proteobacteria* were rich in patients with CRC, and many other researchers have come to the same conclusion, as for the individuals with polyp, principal component analysis shows a significant separation, although the composition of the species did not have such a difference. When the disease progresses to a precancerous stage, during those periods, microbiota seemed to reach a relatively stable and similar situation, in which they have a high degree of similarity to some extent. Above all, also indicated that the microorganisms changed in the early period of precancer and maintained until the later period of precancer, it is the driving role that works at an early stage [9, 34].

In many existing studies, there are also other bacteria to be proved to play an indispensable role across stages of colorectal carcinogenesis, including *Butyricicoccus*, *E. coli* [25, 35], *Parvimonas micra* and *Solobacterium moorei* [26], *Bacteroides fragilis* [27, 36], *Parvimonas micra* and *Peptostreptococcus* [28, 37], *Prevotella* [38], *Campylobacter jejuni* [3], *Faecalibacterium prausnitzii*, *Bifidobacterium*, and *lactobacillus genus* [31].

Another unique feature of our study is that animal experiments are used to confirm that microflora changes indeed promote the occurrence and development of CRC. In Jobin and Furet study [39, 40], fecal bacteria from CRC patients or healthy people were transplanted to sterile and normal mice; the normal mice showed significantly increased hyperatypical hyperplasia and macroscopic polyps, while the cell proliferation of sterile mice increased, but the fecal flora abundance of both types of mice decreased. The study suggests a causal relationship between the bacteria and colorectal cancer, and could lead to new treatments. It is well argued that gavage of fecal samples from patients with colorectal cancer promotes intestinal carcinogenesis in germ-free and conventional mice [41]. Fecal transplantation is widely recognized in the treatment of *C. difficile* infections, it also has potential applications for other diseases, such as fighting against other refractory pathogens under the pressure of antibiotic treatment options. Fecal transplantation may also be considered for use in a variety of chronic diseases under certain off-balance conditions [42]. However, a large number of studies is still needed to prove the method and effect of faecal transplantation.

Our study has certain limitations; we were unable to unravel microecosystems established by specific ones, that may have unknowm coexclusive relationships between members of keystone hypothesis; our gut microbiome studies were based on stool samples, which may reflect the disease state but possibly not the tumor microenvironment, for there is always a lower pH in the tumor environment, and some scholars discovered that a tiny change in pH will cause massive fluctuations in gut microbes, including the genus *Fusobacterium* [25]. The genetic phenotype proved to be associated with the disease but was not investigated in our study. Interindividual variations in the tumorassociated genetic phenotype have posed a long-standing challenge for deciphering microbial signatures implicated in colorectal tumorigenesis.

Last but not least, diet is associated with increased incidence of CRC. Diet shapes the microflora and affects its metabolites and functions. Excessive intake of animal protein and fat (especially red meat and processed meat) will produce excessive secondary bile acid and hydrogen sulfide, leading to barrier dysfunction, inflammation, DNA damage, genotoxicity, and so on, which may increase the risk of CRC. Dietary fiber produces short-chain fatty acids, such as butyric acid. Through cell metabolism, bacterial homeostasis, antiproliferation, immune regulation, and genetic/epigenetic regulation, it plays an anti-inflammatory and antitumor role and protects colon epithelial cells. A balanced diet rich in dietary fiber prevents CRC [6, 43, 44].

## Figures and Tables

**Figure 1:** (a) Venn diagram of OUT and (b) dilution curve of the alpha diversity index. As is shown, the dilution curve of Sobs index with the curve is going to flatten out. (c) Principal component analysis (PCA) based on OTU abundance between groups CC and HC. *x*-axis, 1st principal component and *Y*-axis, 2nd principal component; 14.73% in brackets represents contributions of PC1 components to samples, 10.34% represents contributions of PC2 components to samples. A dot represents each sample, and different colors represent different groups (red: group CC and blue: group HC). (d) OUT rank curve.

**Figure 2:** Alpha diversity indices boxplot between group CC and HC. The abnormal value is shown as “o.”

**Figure 3:** Principal coordinates analysis (PCOA) between group HC and group CC. The figure shows the three-dimensional diagram of PCOA, in which each dot represents a sample, and each color represents a group: red for group CC and blue for group HC. PC1 is the principal coordinate component causing the largest difference in samples, with an explanatory value of 14%. PC2 and PC3 were next, with an explanatory value of 9% and 6%, respectively.

**Figure 4:** The taxonomic composition distribution in samples of the Phylumlevel. Relative abundance of bacterial phyla in microbiota in the healthy control group (HC) and relative abundance of bacterial phyla in microbiota in the CRC group (CC).

**Figure 5:** Proportions of main bacteria of the group CC and HC at the level of phylum (a, b) and genus (c, d). The pie chart of species proportion was obtained by calculating absolute abundance at the phylum and genus level, the major species are selected with a proportional advantage, and the percentage is accurate to 2-3 decimal places.

**Figure 6:** The taxonomic composition distribution in samples of the genus level. Relative abundance of bacterial genus in microbiota in the CRC group (CC) and relative abundance of bacterial genus in the healthy control group (HC).

**Figure 7:** Alpha diversity indices boxplot among four groups. Analysis of the Chao, Sobs, Ace richness index, Shannon index, and Simpson diversity index in A-CC-HC-P groups. (a) Boxplots of the Sobs richness index. (b) Boxplots of the Chao richness index. (c) Boxplots of the Ace richness index. (d) Boxplots of the Shannon diversity index. (e) Boxplots of Simpson diversity index.

**Figure 8:** Principal component analysis (PCA) based on OTU abundance. (a) Group HC and P, PC1 (16.63%) and PC2 (8.65%). (b) Group A and HC, PC1 (16.69%) and PC2 (8.41%).

**Figure 9:** Unweighted UniFrac principal component analysis (PCOA). The microbiota of healthy controls and individuals with polyps (a) as well as healthy controls and individuals with adenoma (b) were significantly different; no difference was found in microbiota composition of individuals with polyps and individuals with adenoma (c).

**Figure 10:** Unweighted UniFrac principal component analysis (PCOA) among groups. Both the 3D images indicate that there does not exist a distinct separation between group A, P (which is considered as precancerous diseases), and group CC.

**Figure 11:** Proportions of main bacteria of the (a) group A and (b) P at the level of phylum.

**Figure 12:** The trend chart based on the main microbial composition for each group at the phylum level. On the phylum level, the abundance of *Bacteroidetes* and *Firmicutes* is decreasing with the development of health-polyp-adenomas-CRC, and the abundance of *Proteobacteria* is increasing.

**Table 1:** Details about exclusion/inclusion criteria.

	Exclusion criteria	Inclusion criteria
(1)	Those who had used antibiotics or microecological agents within 2 months before enrollment	Patients with colorectal cancer/adenoma/polyp who meet the diagnostic criteria and were diagnosed as colorectal cancer/adenoma/polyp by histopathological examination
(2)	Those who currently have intestinal infection or digestive tract symptoms	Without colonoscopy, adjuvant chemoradiotherapy and surgical treatment before sampling
(3)	Those who suffer from chronic diseases such as hypertension, heart disease, and diabetes	Informed consent for this study
(4)	Those who cannot cooperate with major diseases	

**Table 2:** PCR amplification reaction system (20 *μ*L).

The reagents	Volume
5 × PCR buffer	4 *μ*l
2.5 mM dNTP	2 *μ*l
Template NDA	10 ng
5 *μ*M primer	0.8 *μ*l
FastPfu polymerase	0.4 *μ*l
Distilled water	Up to 20 *μ*l

**Table 3:** Richness and diversity analysis.

Alpha diversity	Colorectal cancer	Healthy control	*P* value
index	(*n* = 51)	(*n* = 42)	
Sobs	217.3 ± 69.4	228.8 ± 44.4	0.33
Chao	265.1 ± 80.7	272.9 ± 58.6	0.45
Ace	268.6 ± 78.1	271.9 ± 57.2	0.71
Shannon	2.8 ± 0.8	3.0 ± 0.6	0.2
Simpson	0.2 ± 0.15	0.14 ± 0.1	0.3

**Table 4:** Difference analysis at the phylum level.

Phylum	Mean		*P* value	FDR
	CC	HC		
*Firmicutes*	25.362556	35.878729	0.000356	0.002314
*Fusobacteria*	3.452689	0.596747	0.000001	0.000013
*Proteobacteria*	22.36843	9.325738	0.000796	0.003449
*Spirochaetes*	0.011262	0	0.013421	0.034895
*Synergistetes*	0.193583	0.004467	0.005642	0.018337

**Table 5:** Richness and diversity analysis and proportions of main bacteria at the phylum level.

Index	Healthy group (*n* = 42)	Polyp group (*n* = 59)	Adenoma group (*n* = 54)	CRC group (*n* = 51)
Chao richness index	271.9 ± 58.6	238.4 ± 70.1	240.0 ± 63.2	265 ± 80.7
Shannon index	3.01 ± 0.56	2.72 ± 0.72	2.77 ± 0.59	2.79 ± 0.77
Simpson index	0.14 ± 0.10	0.18 ± 0.13	0.15 ± 0.10	0.17 ± 0.15

Bacteria				
*Bacteroidetes* (%)	52.14	53.92	52.46	47.06
*Firmicutes* (%)	35.88	29.73	24.27	25.36
*Proteobacteria* (%)	9.33	12.31	16.51	22.37
*Fusobacteria* (%)	0.60	1.97	3.98	3.45
*Actinobacteria* (%)	1.25	1.76	1.89	0.72

**Table 6:** Analysis of differences between groups.

	Phylum	*P* value	FDR
A-P	*Fusobacteria*	0.002794	0.039116

A-HC	*Firmicutes*	0.000064	0.000416
	*Fusobacteria*	0	0
	*Proteobacteria*	0.001633	0.007076

CC-HC	*Firmicutes*	0.000356	0.002314
	*Fusobacteria*	0.000001	0.000013

P-HC	*Firmicutes*	0.015437	0.10034
	*Fusobacteria*	0.000625	0.008125

CC-P	*Fusobacteria*	0.012989	0.060615

P-A-CC	*Fusobacteria*	0.004726	0.022055
HC-P-A		0	0.004431
HC-A-CC		0	0

**Table 7:** The eligibility criteria and exclusion criteria for colonoscopy.

*Eligibility criteria for colonoscopy included*
(1) Age of 50–70 years
(2) Absence of existing or previous CRC symptoms, such as haematochezia, tarry stool, change in bowel habit in the past 4 weeks, or a weight loss of 45 kg in the past 6 months
(3) Not having received any CRC screening tests in the past 5 years

*The exclusion criteria for colonoscopy included*
(1) Personal history of CRC, inflammatory bowel disease, prosthetic heart valve, or vascular graft surgery
(2) The presence of medical disorders, which were contraindications for colonoscopy
(3) Those who have used antibiotics or microecological agents within 2 months before enrollment
(4) Those who currently have intestinal infection or digestive symptoms
(5) Those who suffer from chronic diseases such as hypertension, heart disease, and diabetes
(6) Those who cannot cooperate with major diseases
Abbreviations: CRC, colorectal cancer

## Data Availability

The data used to support the findings of this study are included within the article.
